This article has been retracted.

# Dysregulated Circulating Apoptosis- and Autophagy-Related lncRNAs as Diagnostic Markers in Coronary Artery Disease

**DOI:** 10.1155/2021/5517786

**Published:** 2021-08-31

**Authors:** Lijiao Zhang, Dayuan Lou, Dan He, Ying Wang, Yuhang Wu, Xinyang Cao, Peng Qu

**Affiliations:** ^1^Department of Cardiology, The Second Affiliated Hospital of Dalian Medical University, Dalian, 116027 Liaoning, China; ^2^Department of Physiology and Pathophysiology, School of Basic Medical Sciences, Peking University, Beijing 100191, China; ^3^Institute of Heart & Vessel Diseases, The Second Affiliated Hospital of Dalian Medical University, Dalian, 116027 Liaoning, China

## Abstract

**Objective:**

Increasing evidence emphasizes the implications of dysregulated apoptosis and autophagy cellular processes in coronary artery disease (CAD). Herein, we aimed to explore apoptosis- and autophagy-related long noncoding RNAs (lncRNAs) in peripheral blood of CAD patients.

**Methods:**

The mRNA and lncRNA expression profiles were retrieved from the Gene Expression Omnibus (GEO) database. With ∣fold change | >1.5 and adjusted *p* value < 0.05, differentially expressed apoptosis- and autophagy-related mRNAs were screened between CAD and healthy blood samples. Also, differentially expressed lncRNAs were identified for CAD. Using the psych package, apoptosis- and autophagy-related lncRNAs were defined with Spearson's correlation analysis. Receiver operating characteristic (ROC) curves were conducted for the assessment of the diagnosed efficacy of these apoptosis- and autophagy-related lncRNAs.

**Results:**

Our results showed that 24 apoptosis- and autophagy-related mRNAs were abnormally expressed in CAD than normal controls. 12 circulating upregulated and 1 downregulated apoptosis- and autophagy-related lncRNAs were identified for CAD. The ROCs confirmed that AC004485.3 (AUC = 0.899), AC004920.3 (AUC = 0.93), AJ006998.2 (AUC = 0.776), H19 (AUC = 0.943), RP5-902P8.10 (AUC = 0.956), RP5-1114G22.2 (AUC = 0.883), RP11-247A12.1 (AUC = 0.885), RP11-288L9.4 (AUC = 0.928), RP11-344B5.2 (AUC = 0.858), RP11-452C8.1 (AUC = 0.929), RP11-565A3.1 (AUC = 0.893), and XXbac-B33L19.4 (AUC = 0.932) exhibited good performance in differentiating CAD from healthy controls.

**Conclusion:**

Collectively, our findings proposed that circulating apoptosis- and autophagy-related lncRNAs could become underlying diagnostic markers for CAD in clinical practice.

## 1. Introduction

Coronary artery disease (CAD), as a commonly diagnosed heart disease, contributes to the dominant cause of cardiovascular-related deaths [1]. This disease mainly occurs when the myocardial blood supply decreases [2]. It is composed of myocardial infarction and stable and unstable angina, as well as sudden cardiac death [3]. The etiology of CAD remains little understood due to complex causes such as environmental or genetic risk factors [4]. Hence, it requires exploring in depth for the pathogenesis of CAD. Despite much progress in CAD management, the prevalence is still rising and clinical outcomes are unsatisfactory. Currently, the gold standard for diagnosing CAD is still coronary angiography, and a peripheral blood biochemical test is only used for evaluating the risk factors of CAD. Increasing evidence highlights that circulating biomarkers that can be detected in peripheral blood can be applied for early detection in patients with high-risk CAD [5]. The noninvasive early diagnosis may prevent the progression of CAD, thereby validly lowering its mortality [6]. Nevertheless, there is still lack of circulating markers with high diagnostic value for CAD in clinical practice [7].

Apoptosis and autophagy, as two types of programmed cellular deaths, are both involved in the development of CAD [8]. Undue apoptosis inevitably induces cell death under oxidative stress, ischemia conditions, and the like [9]. Meanwhile, autophagy is an evolutionarily conserved cellular process that participates in degrading and recycling the redundant or useless protein constituents, organelles, and the like [10]. This process is fundamental for maintaining intracellular homeostasis. Hence, its disorder in cardiac cells exerts destructive impacts on the cardiovascular system [11]. Currently, activation of autophagy has been a therapeutic approach for heart diseases [12]. Increasing evidence emphasizes the implications of the interplay between autophagy and apoptosis in CAD [13]. The balance between the two decides cell survival. Both serum levels in CAD patients are higher than healthy controls [14]. lncRNAs with >200 nucleotides may participate in the pathophysiological processes of CAD including autophagy and apoptosis [15]. On account of their tissue and cell specificity, circulating lncRNAs are promising diagnostic markers for various diseases [15]. A previous study has identified three lncRNAs including Chast, HULC, and DICER1-AS1 that are distinctly related to autophagy in blood circulation of CAD patients [16]. Among them, HULC and DICER1-AS1 may properly differentiate CAD individuals from healthy individuals. It has been demonstrated that apoptosis and autophagy may be mediated by several common lncRNAs in CAD. For example, lncRNA MALAT1 [17] or THRIL [18] inhibits autophagy and apoptosis of endothelial progenitor cells in CAD. However, it remains unclear what the clinical implications of autophagy- and apoptosis-related lncRNAs in CAD are. Herein, we firstly screened circulating dysregulated apoptosis- and autophagy-related mRNAs in CAD. Secondly, circulating abnormally expressed lncRNAs were identified in CAD compared to healthy subjects. Thirdly, Spearson's correlation analysis was employed for identifying circulating apoptosis- and autophagy-related lncRNAs, and ROC curves were conducted for evaluating their diagnostic efficacy for CAD. Finally, their expression was externally verified in blood specimens of CAD and healthy subjects.  Figure 1 showed the workflow of this study. These lncRNAs proposed by our findings may reflect the pathologically relevant processes that occurred in CAD, which could provide a novel insight into the diagnosis and management of CAD.

## 2. Materials and Methods

### 2.1. Datasets and Preprocessing

The mRNA and lncRNA expression profiles of CAD patients and healthy controls were searched from the Gene Expression Omnibus (GEO; https://www.ncbi.nlm.nih.gov/geo/query/acc.cgi) according to the following criteria: organism—*Homo sapiens*; experiment type—noncoding RNA profiling by array; and disease—CAD. As a result, two datasets including GSE113079 and GSE69587 datasets were obtained for this study. The GSE113079 dataset included 93 CAD and 48 healthy blood samples based on the GPL20115 platform [19]. The GSE69587 dataset was composed of 3 CAD and 3 healthy blood specimens on the platform of GPL15314 [20]. The microarray data were normalized to quartile by the normalizeBetweenArrays in the limma package [21]. If the same gene corresponded to multiple IDs, the average value was calculated as the expression level of the gene.

### 2.2. Differential Expression Analysis

Differentially expressed mRNAs or lncRNAs were screened between CAD and healthy groups with the cutoff of ∣fold change (FC) | >1.5 and adjusted *p* value < 0.05 via the limma package, which were visualized into volcano and heatmaps [21].

### 2.3. Autophagy- and Apoptosis-Related mRNAs

Genes in autophagy (entry: map04140) and apoptosis (entry: map04210) were obtained from the Kyoto Encyclopedia of Genes and Genomes database (KEGG; https://www.kegg.jp/) [22]. They were overlapped by differentially expressed mRNAs called differentially expressed autophagy- and apoptosis-related mRNAs.

### 2.4. Protein-Protein Interaction (PPI)

Physical or functional interactions between specified proteins were analyzed via the STRING online tool (http://string-db.org/) [23]. Required confidence (combined score) > 0.7 was set as the cutoff of the interactions. Cytoscape software was utilized to visualize the PPI network [24]. Connectivity degree was calculated, and hub genes with degree ≥ 3 were obtained [25].

### 2.5. Correlation Analysis

Spearson's correlation analysis between differentially expressed lncRNAs and differentially expressed autophagy- and apoptosis-related mRNAs was presented via the psych package in R. lncRNAs with correlation *p* value < 0.05 with at least 50% of differentially expressed autophagy- and apoptosis-related mRNAs were considered as differentially expressed autophagy- and apoptosis-related lncRNAs.

### 2.6. External Validation

The expression of differentially expressed autophagy- and apoptosis-related lncRNAs was externally verified in blood samples from 5 CAD patients and 5 healthy controls in the GSE169256 dataset. Moreover, associations between their expression and clinical features (age) were analyzed by Spearson's correlation tests. Their expression was also compared between male and female patients.

### 2.7. Statistical Analysis

Based on the expression profiles of the differentially expressed autophagy- and apoptosis-related lncRNAs, relative operating characteristic curves (ROCs) were conducted via the pROC package in R in the GSE113079 dataset [26].

## 3. Results

### 3.1. Circulating Abnormally Expressed mRNAs for CAD

To explore CAD-related mRNAs, we screened abnormally expressed mRNAs between 93 CAD and 48 healthy blood samples in the GSE113079 dataset. Firstly, we normalized the microarray data via the limma package (Figures 2(a) and 2(b)). 988 up- and 831 downregulated mRNAs were obtained in CAD compared to normal samples (Figures 2(c) and 2(d)). The top five upregulated mRNAs included KIF17, BIRC7, TRPM5, NMNAT2, and ACTBL2. The top five downregulated mRNAs were as follows: CSNK1A1, C22orf31, KRT33B, PAK2, and LONRF3. Heatmaps demonstrated that these mRNAs clearly distinguished CAD samples into healthy samples (Figure 2(e)).  Figure 2(f) visualized the top 20 abnormally expressed mRNAs in CAD and healthy blood samples. The details of the top ten up- and downregulated mRNAs were separately listed in Tables 1 and 2. There were distinct differences in their expressions between CAD and healthy samples indicating that they could participate in the progression of CAD.

### 3.2. Abnormally Expressed Autophagy- and Apoptosis-Related mRNAs in CAD

To find autophagy- and apoptosis-related mRNAs in CAD, we overlapped the abnormally expressed mRNAs and autophagy- and apoptosis-related mRNAs. As a result, 24 mRNAs were identified for CAD (Figure 3(a)), as follows: ATG2B, CAPN2, CASP8, CTSW, DFFB, FASLG, GABARAPL1, GZMB, HIF1A, ITPR3, JUN, LMNA, MAPK9, MTMR4, NGF, PIK3R2, PPP2CA, PRF1, PRKACA, RRAGB, RRAS2, TNFSF10, TP53AIP1, and TUBA8. We further analyzed whether the proteins encoded by them had physical or functional interactions. A PPI network was constructed based on them, which was made up of 15 nodes (Figure 3(b)). Among all nodes in the network, PRKACA (degree = 3), TNFSF10 (degree = 2), NGF (degree = 3), PIK3R2 (degree = 1), and TUBA8 (degree = 1) were highly expressed in CAD compared to healthy samples. MAPK9 (degree = 2), JUN (degree = 5), HIF1A (degree = 1), GABARAPL1 (degree = 1), ITPR3 (degree = 1), LMNA (degree = 1), PRF1 (degree = 2), GZMB (degree = 5), FASLG (degree = 5), and CASP8 (degree = 3) were poorly expressed in CAD compared to healthy samples.

### 3.3. Abnormally Expressed Circulating lncRNAs for CAD

Circulating lncRNAs have been considered as diagnosed biomarkers for CAD [27]. Herein, two datasets GSE113079 and GSE69587 were collected for screening abnormally expressed circulating lncRNAs for CAD. In the GSE113079 dataset, we normalized the microarray data of each sample (Figures 4(a) and 4(b)). Then, 1382 up- and 1356 downregulated lncRNAs were identified for CAD blood compared to healthy blood samples (Figure 4(c) and 4(d)). The top five upregulated lncRNAs included RP11-548O1.3, RP11-216N14.9, XLOC_I2_013427, RP11-370I10.2, and linc-SALL1-3. Meanwhile, the top five downregulated lncRNAs covered linc-ID2-3, RP11-689C9.1, linc-ANKRD30A-3, LOC100130865, and MTRNR2L9. CAD samples were distinctly distinguished from healthy samples (Figure 4(e)). The top 20 abnormally expressed circulating lncRNAs were visualized in Figure 4(f).  Table 3 listed the detailed information of the top ten circulating upregulated lncRNAs for CAD in the GSE113079 dataset. Meanwhile, the detailed information of the top ten circulating downregulated lncRNAs for CAD in the GSE113079 dataset is shown in Table 4.

Since the GSE69587 dataset has been standardized, this study no longer standardized the dataset. In total, 430 circulating lncRNAs were upregulated and 305 circulating lncRNAs were downregulated in CAD compared to healthy samples (Figures 5(a) and 5(b)). The top five up- (LOC284440, AK096649, AC118138.2, lincRNA-FYN-1, and RP11-372K14.2) and downregulated lncRNAs (AC005779.1, RP11-474J18.1, LOC400657, AK293020, and BC034788) were listed, respectively. Based on the expression levels of these lncRNAs, CAD samples were distinguished from healthy samples (Figure 5(c)).  Figure 5(d) depicts the top 20 abnormally expressed circulating lncRNAs. To increase the reliability of the results, we overlapped the abnormally expressed lncRNAs in the GSE113079 and GSE69587 datasets. Consequently, 12 upregulated lncRNAs were obtained for CAD, including AC004485.3, AC004920.3, AJ006998.2, H19, RP11-247A12.1, RP11-288L9.4, RP11-344B5.2, RP11-452C8.1, RP11-565A3.1, RP5-1114G22.2, RP5-902P8.10, and XXbac-B33L19.4 (Figure 6(a)). Moreover, LOC338758 was downregulated in CAD blood samples (Figure 6(b)). These lncRNAs could be involved in CAD development.

### 3.4. Abnormally Expressed Autophagy- and Apoptosis-Related Circulating lncRNAs for CAD

We analyzed the correlation between 13 abnormally expressed circulating lncRNAs and autophagy- and apoptosis-related mRNAs. Herein, we found that PRKACA, PIK3R2, and NGF were positively related to the 12 upregulated lncRNAs (all *p* < 0.05; Figure 7 and Supplementary Table 1). TP53AIP1, RRAS2, PRF1, PPP2CA, MTMR4, MAPK9, LMNA, ITPR3, HIF1A, DFFB, CASP8, CAPN2, and ATG2B were negatively correlated to the 12 upregulated lncRNAs (all *p* < 0.05). Meanwhile, JUN and ITPR3 had positive correlations with downregulated LOC338758 (both *p* < 0.05). Thus, these lncRNAs could be distinctly related to autophagy and apoptosis in CAD.

### 3.5. Highly Expressed Autophagy- and Apoptosis-Related Circulating lncRNAs as Diagnostic Markers for CAD

In the GSE113079 dataset, we compared the differences in expression of the 12 upregulated autophagy- and apoptosis-related lncRNAs in CAD and healthy blood samples. Our results showed that 11 lncRNAs were distinctly highly expressed in CAD compared to controls, including AC004485.3 (log 2 FC = 1.048; *p* = 1.32*e*‐25), AJ006998.2 (log 2 FC = 0.607; *p* = 8.14*e*‐10), H19 (log 2 FC = 0.713; *p* = 5.18*e*‐16), RP11-247A12.1 (log 2 FC = 0.622; *p* = 3.15*e*‐17), RP11-288L9.4 (log 2 FC = 0.768; *p* = 1.06*e*‐23), RP11-344B5.2 (log 2 FC = 0.968; *p* = 2.52*e*‐11), RP11-452C8.1 (log 2 FC = 0.87; *p* = 5.3*e*‐24), RP11-565A3.1 (log 2 FC = 0.618; *p* = 1.29*e*‐15), RP5-1114G22.2 (log 2 FC = 0.717; p = 1.26e‐11), RP5-902P8.10 (log 2 FC = 0.79; *p* = 1.2*e*‐32), and XXbac-B33L19.4 (log 2 FC = 0.966; *p* = 4.03*e*‐28; Figure 8). These lncRNAs could be related to CAD progression.

### 3.6. Validation of the Diagnostic Efficacy of Autophagy- and Apoptosis-Related Circulating lncRNAs for CAD

The diagnostic efficacy of the autophagy- and apoptosis-related circulating lncRNAs was assessed via ROCs. The areas under the curves (AUCs) are as follows: AC004485.3 (AUC = 0.899; 95%CI = 0.845‐0.954; Figure 9(a)), AC004920.3 (AUC = 0.93; 95%CI = 0.885‐0.974; Figure 9(b)), AJ006998.2 (AUC = 0.776; 95%CI = 0.691‐0.861; Figure 9(c)), H19 (AUC = 0.943; 95%CI = 0.909‐0.976; Figure 9(d)), RP5-902P8.10 (AUC = 0.956; 95%CI = 0.919‐0.993; Figure 9(e)), RP5-1114G22.2 (AUC = 0.883; 95%CI = 0.827‐0.939; Figure 9(f)), RP11-247A12.1 (AUC = 0.885; 95%CI = 0.828‐0.942; Figure 9(g)), RP11-288L9.4 (AUC = 0.928; 95%CI = 0.881‐0.975; Figure 9(h)), RP11-344B5.2 (AUC = 0.858; 95%CI = 0.789‐0.926; Figure 9(i)), RP11-452C8.1 (AUC = 0.929; 95%CI = 0.885‐0.972; Figure 9(j)), RP11-565A3.1 (AUC = 0.893; 95%CI = 0.824‐0.962; Figure 9(k)), and XXbac-B33L19.4 (AUC = 0.932; 95%CI = 0.888‐0.976; Figure 9(l)). The data above suggested that these lncRNAs accurately differentiated CAD from healthy controls. Thus, these lncRNAs could be underlying circulating diagnostic markers for CAD.

### 3.7. External Validation of Autophagy- and Apoptosis-Related Circulating lncRNAs in CAD

To further verify the expression of autophagy- and apoptosis-related circulating lncRNAs in CAD, we employed the GSE169256 dataset. Spearson's correlation analysis showed that AC004485.3 and AC004920.3 were both negatively correlated to age, while AJ006998.2, H19, LOC338758, RP11-247A12.1, RP11-288L9.4, RP11-452C8.1, RP11-565A3.1, RP5-1114G22.2, RP5-902P8.10, and XXbac-B33L19.4 were positively correlated to age (Figure 10(a)).  Figure 10(b) shows the differences in expression of the above lncRNAs between male and female CAD patients. Furthermore, the abnormal expression of these lncRNAs was externally confirmed by comparing 5 CAD patients and 5 healthy controls in the GSE169256 dataset (Figure 10(c)).

## 4. Discussion

CAD is the most common cause of death globally, which usually kills approximately 17 million individuals each year [28]. Circulating lncRNAs, with tissue and cell specificity, may discern the risk of CAD and assist in formulating therapeutic therapy [29]. In comparison to the conventional diagnosed approach, circulating lncRNAs are noninvasive and innocuous, with highly sensitive and accurate advantages [30]. Furthermore, lncRNAs may participate in the progression of CAD via mediating apoptosis and autophagy, two forms of programmed cell deaths [15]. On account of these strengths, this study explored circulating lncRNAs related to apoptosis and autophagy for CAD diagnosis. However, so far, there is still a lack of circulating lncRNAs for the diagnosis of CAD. To fill the gap, our study identified 12 apoptosis- and autophagy-related circulating lncRNAs that had good performance in diagnosing CAD.

In this study, 988 up- and 831 downregulated mRNAs were screened for CAD compared to healthy controls in blood samples. Among them, KIF17, BIRC7, TRPM5, NMNAT2, ACTBL2, CSNK1A1, C22orf31, KRT33B, PAK2, and LONRF3 had the highest changes in expression between CAD and healthy controls. Among them, a previous study has found that PAK2 activated by METRNL may attenuate cardiomyocyte apoptosis induced by myocardial ischemia/reperfusion [31]. The balance between apoptosis and autophagy exerts a critical role on the pathological conditions of CAD [32]. Among all differentially expressed mRNAs, 24 mRNAs were on the apoptosis and autophagy pathways. Of them, silencing CAPN2 suppresses NF-*κ*B activation as well as decreases myocardial infarction remodeling [33]. CASP8 polymorphic variants (-652 6N del/ins, IVS12-19G>A) could predict the risk of CAD [34]. Furthermore, high CASP8 levels have an association with elevated incidence of coronary diseases [35]. GzmB expression is increased in blood and tissues of CAD patients compared to healthy individuals [34]. H1F1A is significantly altered in CAD patients compared to controls [28]. ITPR3 single-nucleotide polymorphism rs2229634 could be indicative of an increased incidence in coronary artery aneurysm among youngsters [36]. Variants in LMNA are linked with lipodystrophy [37]. Combining previous research, these mRNAs identified by this study may possess tight links to CAD pathogenesis. We constructed a PPI network based on these apoptosis and autophagy mRNAs, which could help to study the pathogenesis of CAD from a systematic perspective. In the network, PRKACA, TNFSF10, NGF, PIK3R2, TUBA8, MAPK9, JUN, HIF1A, GABARAPL1, ITPR3, LMNA, PRF1, GZMB, FASLG, and CASP8 were considered hub genes for CAD. The protein products from these hub genes could have physical and functional associations, which might play vital roles in the biological processes of CAD. In apoptosis and autophagy pathways, the regulation of other genes might be often affected by these hub genes.

Circulating lncRNAs have been proven as diagnosed biomarkers for CAD [19]. By comprehensive analysis of the two datasets, we identified 12 upregulated lncRNAs in CAD compared to controls, including AC004485.3, AC004920.3, AJ006998.2, H19, RP11-247A12.1, RP11-288L9.4, RP11-344B5.2, RP11-452C8.1, RP11-565A3.1, RP5-1114G22.2, RP5-902P8.10, and XXbac-B33L19.4. Moreover, one downregulated lncRNA, LOC338758, was identified in CAD blood samples. These lncRNAs could be involved in CAD progression. Among them, upregulated H19 has been detected in blood samples of CAD patients compared to heathy controls [38]. Other lncRNAs should be explored during CAD development in depth. Considerable research suggests that lncRNAs widely participate in biological processes in CAD, especially apoptosis and autophagy [17, 18, 39]. Here, we analyzed the associations between circulating abnormally expressed lncRNAs and apoptosis- and autophagy-related mRNAs in CAD blood samples. Our data suggested that PRKACA, PIK3R2, and NGF were positively linked to the 12 upregulated lncRNAs. TP53AIP1, RRAS2, PRF1, PPP2CA, MTMR4, MAPK9, LMNA, ITPR3, HIF1A, DFFB, CASP8, CAPN2, and ATG2B had negative correlation to the 12 upregulated lncRNAs. Meanwhile, JUN and ITPR3 exhibited positive relationships with downregulated LOC338758. These data indicated that these lncRNAs could be closely associated with the autophagy and apoptosis processes in CAD.

On account of the shortcomings of current diagnostic markers on CAD, circulating lncRNAs appear to have attracted close attention. After verification, our data demonstrated that AC004485.3 (AUC = 0.899), AC004920.3 (AUC = 0.93), AJ006998.2 (AUC = 0.776), H19 (AUC = 0.943), RP5-902P8.10 (AUC = 0.956), RP5-1114G22.2 (AUC = 0.883), RP11-247A12.1 (AUC = 0.885), RP11-288L9.4 (AUC = 0.928), RP11-344B5.2 (AUC = 0.858), RP11-452C8.1 (AUC = 0.929), RP11-565A3.1 (*A*UC = 0.893), and XXbac-B33L19.4 (AUC = 0.932) exhibited good performance to differentiate CAD from healthy controls. The above findings concerning circulating lncRNAs might possess effective diagnostic value on CAD, thereby reducing mortality. Among them, circulating H19 is correlated to risk of CAD among a Chinese cohort [40]. Additionally, H19 polymorphisms show a tight link to CAD occurrence [41, 42].

Circulating lncRNAs have received much attention in the past years due to their effectiveness and noninvasiveness. This study declared several apoptosis- and autophagy-related circulating lncRNAs with high sensitivity and accuracy. Hence, these lncRNAs might possess the clinical application value as diagnostic markers for CAD, thereby improving the diagnostic accuracy and prolonging patients' survival duration. Several limitations should be considered in this study. First, the conclusion of this study was based on retrospective studies. The diagnostic efficacy of these circulating lncRNAs will be validated in a large-scale, multicenter, and prospective cohort in our future research. Second, the functions of these lncRNAs in apoptosis and autophagy processes are not completely clear in CAD. Their specific mechanisms will be explored in our further experimental studies.

## 5. Conclusion

Collectively, this study identified and externally confirmed that 12 apoptosis- and autophagy-related circulating lncRNAs (AC004485.3, AC004920.3, AJ006998.2, H19, LOC338758, RP11-247A12.1, RP11-288L9.4, RP11-452C8.1, RP11-565A3.1, RP5-1114G22.2, RP5-902P8.10, and XXbac-B33L19.4) were distinctly upregulated in CAD compared to healthy controls. More importantly, they had good performance in distinguishing CAD from healthy individuals. Thus, these circulating lncRNAs could be promising diagnostic markers for CAD.

## Figures and Tables

**Figure 1:** The workflow of this study.

**Figure 2:** Screening circulating abnormally expressed mRNAs for CAD. Box plots for the expression levels of mRNAs in CAD and healthy samples before (a) and after (b) normalization. (c) Scatter and (d) volcano plots for abnormally expressed mRNAs between CAD and healthy samples. (e) Heatmap for the expression patterns of these mRNAs in CAD and healthy samples. (f) Heatmap for the top 20 abnormally expressed mRNAs in CAD and healthy samples. Red: upregulation; blue: downregulation.

**Figure 3:** Identification of abnormally expressed autophagy- and apoptosis-related mRNAs in CAD. (a) Venn diagram for the 24 differentially expressed autophagy- and apoptosis-related mRNAs in CAD. (b) Construction of a PPI network based on them. Red: upregulation; blue: downregulation.

**Figure 4:** Identification of abnormally expressed circulating lncRNAs for CAD in the GSE113079 dataset. Box plots depicting the expression levels of lncRNAs in CAD and healthy samples (a) before and (b) after normalization. (c) Scatter and (d) volcano plots showing all abnormally expressed lncRNAs between CAD and healthy blood samples. (e) Heatmap showing the expression patterns of these lncRNAs in CAD and healthy blood samples. (f) The top 20 abnormally expressed circulating lncRNAs between CAD and healthy groups. Red: upregulation; blue: downregulation.

**Figure 5:** Identification of abnormally expressed circulating lncRNAs for CAD in the GSE69587 dataset. (a) Scatter and (b) volcano diagrams showing abnormally expressed circulating lncRNAs between CAD and healthy samples. (c) Heatmap depicting all abnormally expressed lncRNAs in CAD and healthy blood samples. (d) The top 20 circulating lncRNAs for CAD. Red: upregulation; blue: downregulation.

**Figure 6:** Common abnormally expressed circulating lncRNAs for CAD. (a) 12 upregulated lncRNAs both in the GSE113079 and GSE69587 dataset. (b) One downregulated lncRNA from both the GSE113079 and GSE69587 datasets.

**Figure 7:** Heat map visualizing the correlation between 13 abnormally expressed circulating lncRNAs and autophagy- and apoptosis-related mRNAs in CAD. The color shade represents the absolute value of the correlation coefficient, and the value represents the *p* value. The columns represent lncRNAs, and the rows represent mRNAs.

**Figure 8:** Violin diagram for the expression of 11 circulating lncRNAs in CAD and healthy blood samples, including AC004485.3 (log 2 FC = 1.048; *p* = 1.32*e*‐25), AJ006998.2 (log 2 FC = 0.607; *p* = 8.14*e*‐10), H19 (log 2 FC = 0.713; *p* = 5.18*e*‐16), RP11-247A12.1 (log 2 FC = 0.622; *p* = 3.15*e*‐17), RP11-288L9.4 (log 2 FC = 0.768; *p* = 1.06*e*‐23), RP11-344B5.2 (log 2 FC = 0.968; *p* = 2.52*e*‐11), RP11-452C8.1 (log 2 FC = 0.87; *p* = 5.3*e*‐24), RP11-565A3.1 (log 2 FC = 0.618; *p* = 1.29*e*‐15), RP5-1114G22.2 (log 2 FC = 0.717; *p* = 1.26*e*‐11), RP5-902P8.10 (log 2 FC = 0.79; *p* = 1.2*e*‐32), and XXbac-B33L19.4 (log 2 FC = 0.966; *p* = 4.03*e*‐28).

**Figure 9:** ROC validates 12 circulating lncRNAs as diagnostic markers for CAD: (a) AC004485.3, (b) AC004920.3, (c) AJ006998.2, (d) H19, (e) RP5-902P8.10, (f) RP5-1114G22.2, (g) RP11-247A12.1, (h) RP11-288L9.4, (i) RP11-344B5.2, (j) RP11-452C8.1, (k) RP11-565A3.1, and (l) XXbac-B33L19.4.

**Figure 10:** External validation of autophagy- and apoptosis-related circulating lncRNAs in CAD in the GSE169256 dataset. (a) Spearson's correlation analysis shows the associations between the circulating expression of AC004485.3, AC004920.3, AJ006998.2, H19, LOC338758, RP11-247A12.1, RP11-288L9.4, RP11-452C8.1, RP11-565A3.1, RP5-1114G22.2, RP5-902P8.10, and XXbac-B33L19.4 and age. (b) The differences in expression of the above lncRNAs between male and female CAD patients. (c) External validation of the above lncRNAs in 5 CAD patients and 5 healthy controls.

**Table 1:** The top ten circulating upregulated mRNAs in CAD than healthy controls.

Gene name	Log 2 FC	*p* value	*Q* value	CAD	Healthy
ACTBL2	2.175707163	2.35433*E*‐25	1.3929*E*‐23	2.274988093	0.09928093
BIRC7	1.89222112	2.12792*E*‐36	1.5848*E*‐33	-1.863763605	-3.755984724
KIF17	1.86560487	3.60156*E*‐41	1.51998*E*‐37	-1.141065467	-3.006670337
NMNAT2	1.826600047	4.98533*E*‐31	7.5142*E*‐29	-1.828796794	-3.655396841
TRPM5	1.745508109	1.50641*E*‐34	6.57677*E*‐32	-1.629455661	-3.374963771
NUPR1	1.713797044	2.91563*E*‐34	1.11863*E*‐31	-2.275289877	-3.98908692
AVPR1B	1.628310899	3.45489*E*‐28	3.55629*E*‐26	-1.949760523	-3.578071423
NOG	1.613371937	4.96571*E*‐29	5.56379*E*‐27	0.499062616	-1.114309321
PYDC2	1.604132397	1.92489*E*‐26	1.40873*E*‐24	-2.468823982	-4.072956379
CPEB1	1.548280137	3.14808*E*‐31	5.10998*E*‐29	-2.738597275	-4.286877412

**Table 2:** The top ten circulating downregulated mRNAs in CAD than healthy controls.

Gene name	Log 2 FC	*p* value	*Q* value	CAD	Healthy
KPNA1	-0.585327427	3.78588*E*‐05	9.95082*E*‐05	-3.9803596	-3.395032172
GPRASP1	-0.585805079	4.35625*E*‐10	2.28572*E*‐09	-1.046965965	-0.461160886
RUFY2	-0.585946386	8.90116*E*‐18	1.53958*E*‐16	-0.659711497	-0.073765111
DONSON	-0.586018774	7.67172*E*‐10	3.89149*E*‐09	-1.745995947	-1.159977172
KLHDC1	-0.58626408	3.35774*E*‐09	1.5431*E*‐08	-1.889447587	-1.303183508
MED26	-0.586748565	1.78045*E*‐10	9.89567*E*‐10	-1.114735168	-0.527986603
KDM6A	-0.586918946	3.28334*E*‐09	1.5122*E*‐08	-1.981318284	-1.394399338
SUV39H1	-0.586939293	7.31103*E*‐12	4.96061*E*‐11	-1.621999657	-1.035060363
TAP2	-0.587219549	9.0103*E*‐06	2.59879*E*‐05	0.55477852	1.141998069
FGF7	-0.587788641	3.2713*E*‐07	1.13785*E*‐06	-3.743606566	-3.155817926

**Table 3:** The top ten circulating upregulated lncRNAs for CAD in the GSE113079 dataset.

Gene name	Log 2 FC	*p* value	*Q* value	CAD	Healthy
XLOC_l2_013427	1.983060401	3.43721*E*‐30	6.08964*E*‐28	-2.043809987	-4.026870388
RP11-216N14.9	1.915753591	1.35955*E*‐32	4.462*E*‐30	1.134312816	-0.781440775
RP11-370I10.2	1.850499576	8.17738*E*‐17	1.55324*E*‐15	-2.42064409	-4.271143666
linc-SALL1-3	1.806903286	4.66588*E*‐15	6.86341*E*‐14	-2.027659452	-3.834562738
RP11-548O1.3	1.77753201	3.00599*E*‐34	1.62648*E*‐31	-2.686306726	-4.463838737
RP11-321A17.4	1.725530036	1.14947*E*‐26	9.96205*E*‐25	0.17188431	-1.553645726
CTD-2311B13.1	1.725127268	5.29805*E*‐33	2.12134*E*‐30	-0.390090969	-2.115218237
AC010082.2	1.710990299	9.98176*E*‐38	1.66529*E*‐34	0.180339682	-1.530650617
FAM154A	1.709708154	4.06108*E*‐23	1.93118*E*‐21	-1.554305626	-3.264013779
AC013248.2	1.656964824	1.22892*E*‐19	3.52479*E*‐18	-1.117728421	-2.774693245

**Table 4:** The top ten circulating downregulated lncRNAs for CAD in the GSE113079 dataset.

Gene name	Log 2 FC	*p* value	*Q* value	CAD	Healthy
RP11-689C9.1	-2.635616135	7.33574*E*‐18	1.61386*E*‐16	-0.646839565	1.98877657
MTRNR2L9	-2.223631802	1.54061*E*‐06	6.75198*E*‐06	-2.008594699	0.215037103
linc-ANKRD30A-3	-2.028353512	2.32287*E*‐17	4.76444*E*‐16	0.215910733	2.244264245
LOC100130865	-1.996896907	2.25419*E*‐13	2.62836*E*‐12	-3.03914794	-1.042251032
linc-ID2-3	-1.980200508	6.42151*E*‐24	3.41911*E*‐22	-3.262290981	-1.282090473
RP11-44N11.2	-1.973423235	1.24267*E*‐23	6.26656*E*‐22	-4.09545914	-2.122035905
RP11-464O2.2	-1.896597301	6.03265*E*‐19	1.58288*E*‐17	-3.53754729	-1.640949989
RP4-758J18.7	-1.845072205	8.60858*E*‐11	6.927*E*‐10	-1.180978882	0.664093323
C9orf170	-1.793813177	2.4523*E*‐11	2.15897*E*‐10	-3.381744032	-1.587930855
RP11-214K3.18	-1.770839873	1.37694*E*‐25	1.02097*E*‐23	-2.621810224	-0.850970351

## Data Availability

The data used to support the findings of this study are included within the supplementary information files.

## Abbreviations

CAD: Coronary artery disease
lncRNAs: Long noncoding RNAs
ROC: Receiver operating characteristic
GEO: Gene Expression Omnibus
FC: Fold change
KEGG: Kyoto Encyclopedia of Genes and Genomes database.
PPI: Protein-protein interaction
AUCs: Areas under the curves.

## Supplementary Materials

Supplementary Materials Supplementary Table 1: correlation analysis between 13 abnormally expressed circulating lncRNAs and autophagy- and apoptosis-related mRNAs.
